# Computerized-Assisted Scoliosis Diagnosis Based on Faster R-CNN and ResNet for the Classification of Spine X-Ray Images

**DOI:** 10.1155/2022/3796202

**Published:** 2022-06-06

**Authors:** Peiji Chen, Zhangnan Zhou, Haixia Yu, Kun Chen, Yun Yang

**Affiliations:** ^1^Department of Orthopedics, Huaqiao University Affiliated Strait Hospital, Quanzhou, Fujian 362000, China; ^2^Department of Medical Examination Center, Huaqiao University Affiliated Strait Hospital, Quanzhou, Fujian 362000, China

## Abstract

In order to reduce the subjectivity of preoperative diagnosis and achieve accurate and rapid classification of idiopathic scoliosis and thereby improving the standardization and automation of spinal surgery diagnosis, we implement the Faster R-CNN and ResNet to classify patient spine images. In this paper, the images are based on spine X-ray imaging obtained by our radiology department. We compared the results with the orthopedic surgeon's measurement results for verification and analysis and finally presented the grading results for performance evaluation. The final experimental results can meet the clinical needs, and a fast and robust deep learning-based scoliosis diagnosis algorithm for scoliosis can be achieved without manual intervention using the X-ray scans. This can give rise to a computerized-assisted scoliosis diagnosis based on X-ray imaging, which has strong potential in clinical utility applied to the field of orthopedics.

## 1. Introduction

Adolescent idiopathic scoliosis (AIS) is the most common three-dimensional spinal deformity, accounting for about 80% of the total number of idiopathic scoliosis. In my country, the prevalence of scoliosis is still increasing year by year [1]. The incidence rate among 6-year-old adolescents is 1%-3%, which not only seriously affects the physical appearance of adolescents but also impairs their respiratory function, motor function, mental state, and overall quality of life. In addition, spinal surgery is time-consuming and risky, and the instruments used for surgical correction are complicated, difficult, traumatic, and complicated (major orthopedic surgery). Moreover, the preoperative diagnosis is subjective, which can lead to different diagnoses. Therefore, how to standardize and automate the diagnosis of spine surgery is the significance of this paper.

Generally, orthopedic surgeons manually measure and calculate the Cobb (which relates to the surgeon by the name of John Robert Cobb) angle according to the shape of the spine presented by the X-ray film taken by the patient to determine whether the patient has scoliosis and its severity. Judging from the current research status of the Cobb angle measurement method of scoliosis images, the Cobb angle measurement method has been researched and applied to a certain extent, but more are based on manual and semiautomatic measurement methods proposed for the Cobb angle measurement of scoliosis images. Now, the manual measurement of Cobb angle for scoliosis images still has certain shortcomings and challenges. Notably, manual diagnosis method will increase the workload of the doctor at the same time and waste a large amount of medical resources. With the continuous development of computer hardware and artificial intelligence technology, computer-aided diagnosis based on deep learning has become an important means to assist doctors [2], and certain results have been achieved, which provides a new direction for the medical status of scoliosis diseases. In this paper, we choose X-ray imaging and study the screening method for scoliosis diseases based on the convolutional neural network [3].

## 2. Methods

### 2.1. Target Localization Method Based on Convolutional Neural Network

#### 2.1.1. Faster R-CNN Model (Target Localization Model in the Spine Area) Construction

The Faster R-CNN model [4] consists of two parts: region proposal networks (RPN) and fast region-based convolutional network method (Fast R-CNN). The Faster R-CNN used in this paper obtains the feature map through the basic network structure composed of multiple layers of conv and ReLU (small 5-layer deep ZF network model with low video memory requirements or large 16-layer deep VGG-16 network model with high video memory requirements), and the feature map is shared in the following two parts of the network. The first part is to input the feature map into the RPN to get the region proposal on the feature map. The second part uses Fast R-CNN to classify and accurately locate the region proposal. Finally, the location information and category information of the target can be obtained.  Figure 1 shows the detailed network structure of the spine X-ray image positioning based on Faster R-CNN.

The experimental data used in this paper is the X-ray image of the patient's spine, and the size of the image is 224 × 224 × 3 (3 is the number of channels of the image). A 5-layer deep ZF network is used to extract features, including 5 conv layers, 2 ReLU layers, 2 LRN layers, and 2 maxpool layers. As shown in Figure 1, each conv layer is connected to the ReLU layer, using the ReLU activation function [5].

The basic structure of the first depth of the Faster R-CNN has four layers. The first layer is the conv layer, consisting of 96 7 × 7 × 3 convolution kernels, using stride as 2, padding as 3, and get a result of size 112 × 112 × 96; the second layer is the ReLU layer, and the size of the output result is still 112 × 112 × 96; the third layer is the LRN layer, drawing on the concept of lateral inhibition in biology to achieve local inhibition in the neural network. LRN is used in conjunction with ReLU to enhance pixels with large response, suppress pixels with small response, achieve local normalization, improve the generalization ability of the network, and improve the recognition rate; the fourth layer is the maxpool layer, using a 3 × 3 pooling window, stride is 2, padding is 1, and the size of the output result is 56 × 56 × 96. The structure of the second layer depth of the network is the same as the first depth. The first layer conv layer uses 256 5 × 5 × 3 convolution kernels, stride is 2, padding is 2, and the size of the result is 28 × 28 × 256; the second layer is the ReLU layer; the third layer is the LRN layer; the fourth layer is the maxpool layer, using a 3 × 3 pooling window, stride is 2, padding is 1, and the size of the output result is 28 × 28 × 256. The third layer depth, fourth layer depth, and fifth layer depth of the network have the same structure. They all use the basic conv layer combined with the ReLU layer. The conv layer uses 384, 384, and 256 3 × 3 convolution kernels, respectively, stride is 1, padding is 1, and the depths of the third and fourth layers of the network are both 14 × 14 × 384. The fifth layer depth of the network gets a result with a size of 14 × 14 × 256. Therefore, through the calculation of a simple neural network, a 14 × 14 × 256 feature map is finally obtained.

The RPN is composed of a simple convolutional neural network. First, convolution is performed through 256 3 × 3 convolution kernels to produce a result of 14 × 14 × 256. Then pass two 1 × 1 convolution kernels to form two branches. The first branch is composed of 18 convolution kernels and produces a result of 14 × 14 × 18 (14 × 14 × (9 × 2): 9 anchors, each with two parameters, representing the foreground and background, a total of 18 dimensions). The second branch is composed of 36 convolution kernels and produces a result of 14 × 14 × 36 (14 × 14 × (9 × 4): 9 anchor boxes, each with four parameters, representing the coordinate center, width, and height of the anchor boxes, a total of 36 dimensions). Before entering the ROI Definition network, reshape the result obtained from the first branch (while changing the dimension of the input data without changing the data content) to obtain the required vector.

The RPN is composed of a three-layer network of softmax, reshape, and proposal to generate ROI Definition. Input the 18-dimensional feature vector into softmax to get the probability that each anchor box is foreground and not foreground. After the calculation of this layer is completed, the calculation result is reshaped again to obtain a vector of 14 × 14 × 18. The input of the Definition layer includes the original image (224 × 224 × 3), the vector obtained from the previous layer, and the result obtained by the second branch of the eighth layer depth, as shown in Figure 2. According to the overlap ratio of the real boxes and the predicted boxes, a candidate set of the boxes is generated, and the boxes that exceed the edge and the boxes that do not meet the overlap criterion are discarded.

The R-CNN is composed of ROI pooling, softmax, and four fully connected layers. The feature map and the anchor boxes calculated by the RPN are input to the ROI pooling layer, the feature of the anchor boxes is calculated, and the fully connected layer and the softmax layer are connected. The pooling parameters of this layer are 6 × 6, stride is 6, and the spatial scale is selected to be 1/16 of the original image. The maximum pooling is still selected. Finally, a 6 × 6-dimensional feature vector is obtained. Each anchor area has four parameters, which represent the position information relative to the original image [*x*_1_, *y*_1_, *x*_2_, *y*_2_]. To input the result into the final classification network, only four fully connected layers and one softmax layer are needed. The fully connected layers fc6 and fc7; both use the dropout method to reduce the parameters in the connected layer with a certain probability and reduce the calculation amount of the model [6]. Then connect the fully connected layers boxes_pred and cls_score, respectively. boxes_pred outputs the position information of the precise target box, and cls_score connects the softmax layer to output the probability of the category corresponding to each target, as shown in Figure 3.

The RPN obtains preliminary anchor boxes after passing the IoU restrictions. These anchor boxes cannot correctly detect the position of the target. If you fine-tune the anchor boxes, you can get anchor boxes that are more similar to the ground truth bound so that the frame position information will be more accurate. This paper uses bounding-box regression to fine-tune the anchor boxes. In the current algorithm, input *N* sets of data {(*P*^*i*^, *G*^*i*^)} where *i* = 1, 2, ⋯, *N*, of which *P*^*i*^ = (*P*_*x*_^*i*^, *P*_*y*_^*i*^, *P*_*w*_^*i*^, *P*_*h*_^*i*^), *G*^*i*^ = (*G*_*x*_^*i*^, *G*_*y*_^*i*^, *G*_*w*_^*i*^, *G*_*h*_^*i*^). As shown in Figure 4, *G* represents the ground truth bound, and *P* represents the anchor boxes filtered out.

The idea of bounding-box regression is to input the four values of *G* = (*G*_*x*_, *G*_*y*_, *G*_*w*_, *G*_*h*_) of the ground truth bound and the four values of *P* = (*P*_*x*_, *P*_*y*_, *P*_*w*_, *P*_*h*_) of the anchor boxes to represent the center coordinates, width, and height of the input box and continue to learn to find the appropriate function *f* so that (*G*_*x*_, *G*_*y*_, *G*_*w*_, *G*_*h*_) = *f*(*P*_*x*_, *P*_*y*_, *P*_*w*_, *P*_*h*_) and make the prediction window $\hat{G}$ as close to the real window *G* as possible. Four transformation methods *d*_*x*_(*P*), *d*_*y*_(*P*), *d*_*w*_(*P*), *d*_*h*_(*P*) are used, where *d*_*x*_(*P*), *d*_*y*_(*P*) refer to the translation of the center position without changing the scale, and *d*_*w*_(*P*), *d*_*h*_(*P*) are the translation of the width and height of the specified anchor boxes. Mainly by learning Equation (1), the network translates and zooms the screened anchor boxes to obtain the position information of the prediction window $\hat{G}$.

(1) $$\begin{array}{c} \left\{\begin{array}{c} {\hat{G}}_{x}=P_{w}d_{x}\left(P\right)+P_{x},\\ {\hat{G}}_{y}=P_{h}d_{y}\left(P\right)+P_{y},\\ {\hat{G}}_{w}=P_{w}\exp\left(d_{w}\left(P\right)\right),\\ {\hat{G}}_{h}=P_{h}\exp\left(d_{h}\left(P\right)\right). \end{array}\right. \end{array}$$

In Equation (1), *d*_∗_(*P*) = *w*_∗_^*T*^*φ*(*P*) where ∗ represents *x*, *y*, *w*, *h*. When the anchor boxes are close to the ground truth bound, they can become a linear function to achieve regression. The objective function of the regression is defined according to the training data (*P*, *G*). As in Equation (2), the translation scale and scaling scale (*t*_*x*_, *t*_*y*_, *t*_*w*_, *t*_*h*_) of the optimized model can be obtained.

(2) $$\begin{array}{c} \left\{\begin{array}{c} t_{x}=\frac{\left(G_{x}-P_{x}\right)}{P_{w}},\\ t_{y}=\frac{\left(G_{y}-P_{y}\right)}{P_{h}},\\ t_{x}=\log\left(\frac{G_{w}}{P_{w}}\right),\\ t_{h}=\log\left(\frac{G_{h}}{P_{h}}\right). \end{array}\right. \end{array}$$

Linear regression is *Y* = *WX*, input vector *X*, and continuously learn parameter *W* so that output *Y*′ is constantly close to the true value *Y*. In *d*_∗_(*P*) = *w*_∗_^*T*^*φ*(*P*)(∗represents *x*, *y*, *w*, *h*) in this paper, *φ*(*P*) is the linear feature vector obtained by convolution operation, and *w*_∗_ is a vector used to represent the parameters that can be learned in the model. The calculation formula of *w*_∗_ is Equation (3), which is learned by the least square method of optimization regularization.

(3) $$\begin{array}{c} w_{*}=\underset{{\hat{w}}_{+}}{\arg\min}\overset{N}{\underset{i}{\sum }}{\left(t_{*}^{i}-{\overset{\wedge }{w}}_{*}^{T}\phi \left(P^{i}\right)\right)}^{2}+\lambda {\left\|{\overset{\wedge }{w}}_{*}\right\|}^{2}. \end{array}$$

For the Faster R-CNN training method, this paper uses a 5-layer ZF network and adopts the 4-step alternating training method to train the spine images of patients with scoliosis. Such a method can optimize training parameters and improve network efficiency. The training process of the entire Faster R-CNN can be divided into four stages, as shown in Figure 5.

1. Use the first 5 layers of basic network (conv+ReLU) in the ZF network model to extract the required feature map to train the RPN 1 network model of stage 1
2. Still use the first 5 layers of the basic network (conv+ReLU) in the ZF network model, but use the output of the RPN 1 network model (region proposal) as the input of the training network, and train the Fast R-CNN 1 network model of stage 1. At this stage, RPN and Fast R-CNN do not share convolutional layers
3. Use the Fast R-CNN 1 network parameters of stage 1 to reinitialize the RPN model, fine-tune the unique network layer in RPN, and generate the RPN 2 network model of stage 2. In this way, the two networks of RPN and Fast R-CNN can share the convolutional layer and reduce the number of parameters
4. Fix the shared convolutional layer, and merge the PRN 2 network model generated by stage 2 with the unique layer in the Fast R-CNN model to form a unified network. Continuous iteration, fine-tuning the unique parameters of the Fast R-CNN model, and finally generating the required target positioning model

#### 2.1.2. ResNet Model (Grading Screening Model for Scoliosis Disease) Construction

The ResNet (residual network) convolutional neural network consists of 5 groups of convolutions. Since the number and parameters of each group of convolutions are different, a ResNet convolutional neural network with different layers is formed. There are five forms: ResNet18, ResNet34, ResNet50, ResNet101, and ResNet152. As shown in Figure 6, all ResNet convolutional neural networks include three main parts: the input part, the convolution part of each stage in the middle (the blue box in the figure contains four stages from Conv2_x to Conv5_x), and the output part. Although there are different variants of ResNet convolutional neural networks, they basically follow the structural characteristics shown in the figure. The number of network layers is different, mainly because of the differences in the number of convolutional parameters and building block parameters in the middle groups.

As shown in Figure 6, the input part of the ResNet convolutional neural network is composed of conv layer, batch normalization (batch norm, BN) layer, ReLU layer, and maxpool layer. The experimental data used in this paper is the medical image of the patient's spine area generated by the Faster R-CNN. The size of the image is 128 × 128 × 3 (3 is the number of image channels). The first layer of the input part is the conv layer, which is composed of 64 7 × 7 × 3 convolution kernels, using stride as 2, padding as 3, and getting a result of size 65 × 65 × 64; the second layer is the BN layer, called the batch normalization layer, which can accelerate the convergence speed of the network, improve the gradient dispersion in the network, and prevent the network from overfitting. It is generally used after the convolutional layer; the third layer is the ReLU layer, and the output result is still 65 × 65 × 64; the fourth layer is the maxpool layer, using a 3 × 3 pooling window, stride is 2, no padding, and the output result is 32 × 32 × 64.

The second to fifth depths of the network are composed of different numbers of building blocks. Different numbers of building blocks can form convolution operations of different depths (as shown in Figure 7, the four stages of convolution operations in the blue box). The data in the red box in Figure 7{2, 2, 2, 2}, {3, 4, 6, 3}, {3, 4, 6, 3}, {3, 4, 23, 3}, and {3, 8, 36, 3} are the repeated stacking times of building blocks in ResNet18, ResNet34, ResNet50, ResNet101, and ResNet152, respectively. For example, ResNet50 is composed of an input layer, each module from Conv2_x to Conv5_x corresponding to {3, 4, 6, 3} repeated stacking, and the final output layer (calculation process: 1 + 3 × 3 + 3 × 4 + 3 × 6 + 3 × 3 + 1 = 50). As you can see in Figure 7, there are two different forms of building blocks (purple boxes in the figure). They are the two-layer computing building block in ResNet18 and ResNet34 and the three-layer computing building block in ResNet50, ResNet101, and ResNet152.

Figure 8 shows the detailed structure diagram of different building blocks. Figure 8 (left) shows the original building block structure. The input feature map is divided into two data streams. One data stream undergoes two 3 × 3 convolution operations. After the first layer of convolution operation, there is a ReLU operation. The number of convolution kernels is 64. The stride is 1, the padding is 1, and the output result is 32 × 32 × 64. The other data stream is the input data, 32 × 32 × 64; both have the same dimension and can be added directly across two levels so that the ReLU calculation can be output to the next building block structure. Figure 8 (right) shows that the building block structure introduces 1 × 1 convolution. Through the 1 × 1 convolution operation, the feature map can be arbitrarily increased or reduced in dimension while keeping the size of the feature map unchanged, which reduces the complexity of the convolution operation. The input feature map is still divided into two data streams. One data stream is subjected to three-layer convolution operations. The first layer is 64 1 × 1 convolution kernels, using stride as 1, no padding, and the output result is 32 × 32 × 64. Then, perform a ReLU operation; the second layer is 64 3 × 3 convolution kernels, using stride as 1, padding as 1, and the output result is 32 × 32 × 64, performing a ReLU operation; the third layer is 256 1 × 1 convolution kernels, using stride as 1, no padding, and the output result is 32 × 32 × 256. The other data stream is the input data. After 256 1 × 1 convolution cores, the original 32 × 32 × 64 is upgraded so that the data dimensions in the two data streams are the same, and they are directly added across three levels to perform ReLU calculations. Then, these are output to the structure of the next building block.

#### 2.1.3. Stochastic Gradient Descent Method in ResNet Model

In the ResNet convolutional neural network, the method of batch stochastic gradient descent [7] is generally selected for training. In this way, it is possible to avoid gradient oscillations or falling into local optimal conditions to a certain extent. In ResNet convolutional neural network, the objective function is generally concave function. The gradient descent algorithm is to find the smallest point in the concave function through continuous calculation. Derivatives are very useful for maximum or minimum problems in functions. For the function *y* = *f*(*x*), the derivative is denoted as *f*′(*x*). Use a sufficiently small *ε* to make *f*(*x* − *ε*sign(*f*′(*x*)) smaller than *f*(*x*), so move a small step in the opposite direction of the derivative to reduce *f*(*x*). This technique is gradient descent. The gradient descent method used in this paper is the stochastic gradient descent algorithm. Its core idea is to randomly select a small sample of *B* = {*x*^(1)^, ⋯, *x*^(*m*′)^} from the training set, and the value of *m*′ is generally small. When the entire training set *m* grows, *m*′ is fixed. In this way, only *m*′ samples are needed for each update, which greatly reduces the computational cost of a large training set. The calculation process of the gradient is Equation (4). The calculation process of stochastic gradient descent is Equation (5), where *ε* is the learning rate.

(4) $$\begin{array}{c} g=\frac{1}{m^{\prime }}\nabla_{\theta }\overset{m^{\prime }}{\underset{i=1}{\sum }}L\left(x^{\left(i\right)},y^{\left(i\right)},\theta \right), \end{array}$$

(5) $$\begin{array}{c} \theta ⟵\theta -\varepsilon g. \end{array}$$

### 2.2. Patient's Spine Image Data and Screening

The X-ray images of the patient's spine used in this paper were collected over a period of nearly 3 years from 2019 to 2021. There are two different labels for scoliosis screening data. One is used as a four-classification model for scoliosis disease, as shown in Figure 9, including no disease (Cobb angle is 0°-10°), mild scoliosis (Cobb angle is 11°-25°), moderate scoliosis (Cobb angle is 26°-45°), and severe scoliosis (Cobb angle > 45°) [8], as shown in Table 1. The other is based on the actual needs of patients with scoliosis, with three levels of two categories. Among them, the binary classification model of scoliosis disease is to check whether the patient is sick; the binary classification model of mild scoliosis disease is to check whether the patient has mild scoliosis disease; the binary classification model of severe scoliosis disease is to judge whether the patient has severe scoliosis disease, as shown in Figures 10–12. In this paper, in order to effectively judge the degree of scoliosis in patients, a large number of comparative experiments have been carried out, and different experimental data have been used. A total of 6834 X-ray images of the patient's spine were used in this paper. After preprocessing the data, excluding duplicate data and poor quality data, there are a total of 3600 experimental data.

In order to have all the data used as the training set and test set, increase the reliability of the model, improve the generalization ability of the model, and avoid problems such as overfitting of the model; the experiments in this paper adopt the fourfold cross-validation method for training and testing. Fourfold cross-validation [9–14] refers to the use of the nonrepetitive sampling method in simple random sampling to divide the entire data into four parts; each of which three parts is selected for training the model, and the other one is used for testing the model. In this way, four model training can be performed, four models can be obtained, and four sets of test results can be obtained.

Verification of the target positioning of the spine area is shown in Table 2. In the table, no disease, mild scoliosis disease, moderate scoliosis disease, and severe scoliosis disease [15–19] are represented by 1, 2, 3, and 4, respectively. Model 1, Model 2, Model 3, and Model 4 are four models generated by the fourfold cross-validation.

In order to verify the scoliosis classification screening experiment, the training data and test data distribution of the scoliosis disease binary classification model, mild scoliosis disease binary classification model, and severe scoliosis disease binary classification model is shown in Tables 3–5. In the table, no disease, mild scoliosis disease, moderate scoliosis disease, and severe scoliosis disease are represented by 1, 2, 3, and 4, respectively. Model 1, Model 2, Model 3, and Model 4 are four models generated by the fourfold cross-validation.

### 2.3. Classic Feature Extraction Method and SVM Classifier

In order to make the experiment more convincing, this paper uses traditional machine learning methods and Support Vector Machine (SVM) classifiers as comparative experiments to verify the effect of using Faster R-CNN and ResNet convolutional neural network in the grading experiment of scoliosis disease. This experiment uses the feature extraction of the texture feature and Local Binary Pattern (LBP) to detect the region of interest and uses the SVM classifier to classify scoliosis disease in detail.

Texture feature is used to describe the relationship between different pixels in an image. This paper uses the calculation of a single point pixel and its surrounding point pixels to extract the texture features of the image.

Local Binary Pattern (LBP) can describe the local texture features of the image and extract the local features of the image through different LBP operators. This paper uses the traditional LBP calculation method, defines a 3 × 3 window, sets the gray value of the center of the window as a threshold, and compares the gray values of the 8 pixels around the center with it. If the pixel value is greater than the center, it is marked as 0; otherwise, it is marked as 1. In this way, an 8-bit binary number can be obtained, that is, the LBP code of the center pixel (usually the 8-bit binary code is converted to a decimal code). This paper uses the decimal code of the center pixel to reflect texture information and complete feature extraction.

Support Vector Machine (SVM) is a binary classification classifier commonly used in machine learning. Using this method, this paper fits three binary classification problems of scoliosis disease. In a specific data set, manually label positive and negative samples, find a hyperplane, separate two different types of samples as much as possible, and find the optimal decision surface for data classification. For the binary classification problem of medical images, this paper uses Receiver Operating Characteristic (ROC) curve and Area Under the Curve (AUC) to evaluate the pros and cons of the binary classification classifier. The data can be divided into positive samples and negative samples. In the binary classification model of scoliosis disease, there is scoliosis disease, which is called positive, and there is no scoliosis disease, which is called negative. In the actual data detection process, four situations will occur, as shown in Table 6.

Sensitivity can also be called recall rate or true positive rate (TPR). The specificity is the proportion of all samples without scoliosis that are predicted to be free of scoliosis. The abscissa of the ROC curve is FPR, which is the proportion of all samples without scoliosis that are predicted to have scoliosis. The ordinate of the ROC curve is TPR, which is the proportion of all samples with scoliosis that are predicted to have scoliosis and actually have scoliosis. Ideally, it is expected that FPR is 0 and TPR is 1. If the value of AUC is 1, it is an ideal classifier, and the classification effect is perfect. Therefore, the closer the AUC value is to 1, the better the classification effect. The calculation process of the main evaluation indicators is shown in Table 7.

## 3. Results

Figure 13 shows the four-level labels of the scoliosis screening data, which are operated spine, mild scoliosis, moderate scoliosis, and severe scoliosis.

For the binary classification model of scoliosis disease, from the overall point of view of image classification, the combination of Faster R-CNN and ResNet convolutional neural network has the best classification effect. The AUC value is 0.9087, which fully illustrates that the combination of Faster R-CNN and ResNet convolutional neural network has a better classification effect on scoliosis diseases than traditional machine learning methods. The texture features of the image are TX, combined with the SVM classifier, and a good classification result is also obtained, with an AUC value of 0.8553. The combination of LBP and SVM classifier has the worst effect, with an AUC value of 0.8142.

In Figure 14, for the binary classification model of mild scoliosis disease, the combination of Faster R-CNN and ResNet convolutional neural network has the best classification effect, with an AUC value of 0.8659. The TX of the image combined with the SVM classifier also got a good classification result, with an AUC value of 0.8884. The combination of LBP and SVM classifier has an AUC value of 0.8432.

For the binary classification model of severe scoliosis disease, the combination of Faster R-CNN and ResNet convolutional neural network has the best classification effect, and the AUC value is 0.8603. The combination of LBP and SVM classifier also got a good classification result, with an AUC value of 0.8316. The TX of the image, combined with the SVM classifier, has the worst effect, with an AUC value of 0.8219.

It can be seen from Tables 8–10 that the binary classification model of scoliosis disease, the binary classification model of mild scoliosis, and the binary classification model of severe scoliosis using Faster R-CNN combined with ResNet convolutional neural network are better than using traditional feature extraction combined with SVM classifier in terms of accuracy, sensitivity, and specificity.

## 4. Discussion

In this paper, we use the method of combining traditional feature extraction and SVM classifier to conduct comparative experiments. Analysis of the experimental results shows that the combination of Faster R-CNN and ResNet50 convolutional neural network has a better screening effect for scoliosis diseases. The final experimental results can meet clinical needs.

At present, the preoperative diagnosis of Lenke [20–24] type surgery for idiopathic scoliosis in major domestic hospitals is performed by doctors observing the patient's spine X-rays, using markers and rulers to manually measure the Cobb angle for diagnosis. Different doctors may have deviations in the observation results, and the angle of measurement will also change, so there will be errors between observers. However, the same doctor may have different measurement results every time the same patient is measured, so there are errors within the observer. The error between the observer and the observer affects the accuracy of the operation. The main reason is that the angle is manually measured. In order to replace the doctor in the Cobb angle measurement and classification, to achieve accurate and rapid classification of idiopathic scoliosis, this paper uses a popular deep learning framework and validates and analyzes the results measured by doctors under the test set and shows the classification results. The final experimental results can meet clinical needs. A new algorithm for scoliosis diagnosis based on deep learning that is fast and robust without manual definition is obtained. Note that predictive control algorithms [25, 26] can be used to improve medical image diagnostics and facilitate treatment procedures.

## 5. Conclusion

This paper includes two parts: the location of the region of interest in the X-ray image of the patient's spine and the detailed classification of scoliosis disease using X-ray imaging. In the study of locating the region of interest in the upright image of the patient's spine, this paper chooses the Faster R-CNN convolutional neural network to locate the patient's spine region. In the grading study of scoliosis diseases, this paper first combines the clinical experience of orthopedics experts and divides the patients into four grades according to the size of the Cobb angle of the spine. At the same time, the ResNet convolutional neural network is used to classify scoliosis diseases in detail, and then, the network is optimized. Finally, this paper compares the convolutional neural network method and the classic feature extraction method in machine learning (texture composite features, local binary mode) with the combination of Support Vector Machine (SVM) method, which increases the reliability of the model and improves the generalization ability of the model. From the research results, the combination of Faster R-CNN and three ResNet binary classification models studied in this paper can be used as a reference for orthopedic surgeons to diagnose scoliosis diseases.

## Figures and Tables

**Figure 1:** Network structure diagram of spine image positioning based on Faster R-CNN.

**Figure 2:** The relationship between the input image and the feature map.

**Figure 3:** The expression of anchor boxes in the CT image.

**Figure 4:** Schematic diagram of border regression.

**Figure 5:** Faster R-CNN training process diagram.

**Figure 6:** Scoliosis hierarchical network structure diagram based on ResNet.

**Figure 7:** ResNet structure details.

**Figure 8:** Detailed structure diagrams of different building blocks.

**Figure 9:** Four-classification model for scoliosis disease.

**Figure 10:** Binary classification model of scoliosis disease.

**Figure 11:** Binary classification model of mild scoliosis disease.

**Figure 12:** Binary classification model of severe scoliosis disease.

**Figure 13:** Classification of scoliosis by Faster R-CNN and ResNet.

**Figure 14:** ROC curve of (a) nonsevere and (b) severe scoliosis disease binary classification model comparison experiment.

**Table 1:** Statistical table of samples of X-ray images of the patient's spine.

Cobb angle	Category	Number of samples	Label
0°~10°	No disease	991	1
11°~25°	Mild scoliosis disease	890	2
26°~45°	Moderate scoliosis disease	820	3
>45°	Severe scoliosis disease	899	4

**Table 2:** Faster R-CNN fourfold cross-validation data allocation table.

Faster R-CNN model	Model 1	Model 2	Model 3	Model 4
Target	Spine	Spine	Spine	Spine
Number of samples in the training set (sample label)	2700 (2, 3, 4)	2700 (1, 3, 4)	2700 (1, 2, 4)	2700 (1, 2, 3)
Number of samples in the test set (sample label)	900 (1)	900 (2)	900 (3)	900 (4)

**Table 3:** Fourfold cross-validation data allocation table for scoliosis disease binary classification.

Scoliosis disease binary classification ResNet50 model	Model 1 (1982)	Model 2 (1982)	Model 3 (1982)	Model 4 (1982)
Number of samples in the training set (1/2 sample size) (3/4 sample size)	1534 (768/322) (322/322)	1537 (768/323) (323/323)	1537 (768/323) (323/323)	1538 (769/323) (323/323)
Number of samples in the test set (1/2/3/4 sample size)	448 (223/75/75/75)	445 (223/74/74/74)	445 (223/74/74/74)	444 (222/74/74/74)

**Table 4:** Fourfold cross-validation data allocation table for mild scoliosis disease binary classification.

Mild scoliosis disease binary classification ResNet50 model	Model 1 (1780)	Model 2 (1780)	Model 3 (1780)	Model 4 (1780)
Number of samples in the training set (2/3/4 sample size)	1384 (692/346/346)	1384 (692/346/346)	1385 (693/346/346)	1387 (693/347/347)
Number of samples in the test set (2/3/4 sample size)	396 (198/99/99)	396 (198/99/99)	395 (197/99/99)	393 (197/98/98)

**Table 5:** Fourfold cross-validation data allocation table for severe scoliosis disease binary classification.

Severe scoliosis disease binary classification ResNet50 model	Model 1 (1719)	Model 2 (1719)	Model 3 (1719)	Model 4 (1719)
Number of samples in the training set (3/4 sample size)	1339 (640/699)	1339 (640/699)	1339 (640/699)	1340 (640/700)
Number of samples in the test set (3/4 sample size)	380 (180/200)	380 (180/200)	380 (180/200)	379 (180/199)

**Table 6:** Actual testing situation table.

True positive (TP)	Predicted scoliosis disease and actual scoliosis disease
False positive (FP)	Predicted scoliosis disease and actually no scoliosis disease
True negative (TN)	Predict no scoliosis disease and actually no scoliosis disease
False negative (FN)	Predict no scoliosis disease and actually have scoliosis disease

**Table 7:** Main evaluation indicators.

Sensitivity TPR	$\frac{\text{TP}}{\text{TP}+\text{FN}}$
Specificity TNR	$\frac{\text{TN}}{\text{FP}+\text{TN}}$
FNR	$\frac{\text{FN}}{\text{TP}+\text{FN}}$
FPR	$\frac{\text{FP}}{\text{FP}+\text{TN}}$
Precision	$\frac{\text{TP}}{\text{TP}+\text{FP}}$

**Table 8:** Quantitative index results of scoliosis disease binary classification model.

	Faster R-CNN+ResNet	TX+SVM	LBP+SVM
Precision	0.9132	0.7554	0.7123
Sensitivity	0.8722	0.7426	0.6721
Specificity	0.9140	0.7856	0.8576

**Table 9:** Quantitative index results of mild scoliosis disease binary classification model.

	Faster R-CNN+ResNet	TX+SVM	LBP+SVM
Precision	0.8693	0.7780	0.7397
Sensitivity	0.8415	0.7540	0.6902
Specificity	0.9336	0.7461	0.7373

**Table 10:** Quantitative index results of severe scoliosis disease binary classification model.

	Faster R-CNN+ResNet	TX+SVM	LBP+SVM
Precision	0.8243	0.7545	0.7784
Sensitivity	0.8604	0.7212	0.7203
Specificity	0.9352	0.7853	0.8839

## Data Availability

Data are available on request from the authors due to privacy/ethical restrictions.
